# Classification and Segmentation Algorithm in Benign and Malignant Pulmonary Nodules under Different CT Reconstruction

**DOI:** 10.1155/2022/3490463

**Published:** 2022-04-21

**Authors:** Zhiqian Lu, Feixiang Long, Xiaodong He

**Affiliations:** ^1^Department of Radiology, The People's Hospital of Xuancheng City, Anhui 242000, China; ^2^Cancer Center, Department of Radiology, Zhejiang Provincial People's Hospital (Affiliated People's Hospital, Hangzhou Medical College), Hangzhou 310014, China

## Abstract

**Methods:**

The imaging data of 55 patients with chest CT plain scan in the Xuancheng People's Hospital were collected retrospectively. The data of each patient included lung window reconstruction, mediastinum reconstruction, and bone window reconstruction. The depth neural network and 3D convolution neural network were used to construct the model and train the classification and segmentation algorithm. The pathological results were the gold standard for benign and malignant pulmonary nodules. The classification and segmentation algorithms under three CT reconstruction algorithms were compared and analyzed by analysis of variance.

**Results:**

Under the three CT reconstruction algorithms, the classification accuracy of pulmonary nodule density types was 98.2%, 96.4%, and 94.5%, respectively. The Dice coefficients of all nodule segmentation were 80.32% ± 5.91%, 79.83% ± 6.12%, and 80.17% ± 5.89%, respectively. The diagnostic accuracy between benign and malignant pulmonary nodules under different reconstruction algorithms was 98.2%, 96.4%, and 94.5%, respectively. There was no significant difference in the classification accuracy, Dice coefficients, and diagnostic accuracy of pulmonary nodules under three different reconstruction algorithms (all *P* > 0.05).

**Conclusion:**

The depth neural network algorithm combined with 3D convolution neural network has a good efficiency in identifying benign and malignant pulmonary nodules under different CT reconstruction classification and segmentation algorithms.

## 1. Introduction

The mortality of lung cancer ranks first in the world. It is one of the most malignant tumors threatening human health. For lung cancer, only early diagnosis and treatment can reduce mortality and prolong the survival time of patients [1–4]. Malignant pulmonary nodules often indicate the deterioration of disease progression, and more active and targeted treatment is needed to prevent the continuous deterioration of the disease. Therefore, accurate classification of benign and malignant pulmonary nodules can be an excellent adjuvant treatment of patients' diseases. High-resolution CT is the most commonly used means to detect pulmonary nodules accurately. With the more extensive application of high-resolution CT, the diagnostic burden of imaging doctors is increasing [5, 6]. Inexperienced imaging doctors are more likely to miss diagnosis and misdiagnosis.

In recent years, artificial intelligence (AI) technology has been widely used in various industries [7–9]. The application of AI-aided diagnosis system based on deep learning in imaging diagnosis of pulmonary nodules has made rapid progress, and the early lung cancer detection rate has been improved [10–12]. Applying AI technology to screen massive CT images and mark suspicious nodule lesions preliminarily can help imaging doctors in tertiary hospitals, reduce workload, and improve diagnostic accuracy. This technology can also help grassroots imaging doctors and reduce the missed diagnosis rate of nodules [13].

CT imaging quality is affected by many factors, including radiation dose, reconstruction layer thickness, and reconstruction algorithm [14]. The early identification of benign and malignant pulmonary nodules can help doctors accurately diagnose and take appropriate clinical treatment measures. Therefore, this study intends to design a pulmonary nodule classification and segmentation algorithm which can be stable under different reconstruction algorithms. The 3D convolution neural network is used to mine the pulmonary nodules' imaging features fully. The recursive neural network integrating attention mechanism is used to effectively utilize pulmonary nodules' global and local context information [15, 16]. The two classification and segmentation tasks are used for joint learning, which complement each other to help the model further improve the effect to distinguish and evaluate the benign and malignant pulmonary nodules more accurately.

## 2. Material and Methods

### 2.1. General Data

A total of 55 patients with chest CT examinations in the Xuancheng People's Hospital from October 2018 to December 2020 were collected retrospectively, including 23 males and 32 females, aged 56.07 ± 10.09 years. Inclusion criteria: (1) pulmonary nodules were found; (2) chest CT plain scan images include three reconstruction algorithms: lung window reconstruction, mediastinum reconstruction, and bone reconstruction. Exclusion criteria: (1) excessive respiratory motion artifacts affect CT quality; (2) multiple pulmonary nodules.

### 2.2. Instruments and Methods

GE (Optima CT670) 64 slice spiral CT is adopted: tube voltage 120 kV, tube current 39 mAs, pitch 0.8 and layer thickness 5 mm; Philips (Brilliance) 16 slice spiral CT scanning: tube voltage 120 kV, tube current automatic adjustment, pitch 1, layer thickness 5 mm; the scanning range was from the upper edge of the sternoclavicular joint to the bottom of the lung and breath-holding scanning at the end of inhalation. The images of lung window reconstruction, mediastinum reconstruction, and bone window reconstruction were evaluated.

### 2.3. Construction of Pulmonary Nodule Model

Our study started with the features extracted from the model to build an algorithm model with a long-lasting effect. Multiple steps were used to enhance the features' representation ability and resist the impact of the change in the reconstruction algorithm. The specific framework of the model was shown in Figure 1.

The model design mainly starts from the following four points:

1. Deep neural network is used instead of traditional machine learning to automatically learn features in a data-driven way to avoid the limitations of defining features based on rules in conventional machine learning
2. Compared with the 2D convolutional neural network commonly used in natural images, the 3D convolutional neural network in this study can capture more spatial context information of pulmonary nodules
3. A recurrent neural network with an attention mechanism is constructed, and the 3D convolution neural network replaces the matrix multiplication in the recurrent neural network. The process of subfocus observation of different regions of nodules in daily film reading is modeled as a time-series process by a recurrent neural network. Through continuous iteration, an attention map is generated at each iteration time, different local detail features of nodules are extracted, and multiregion features are fused
4. The upper design of the model adopts the method of multitask learning to predict the nodule contour and the nodule density type simultaneously. In this way, the two tasks complement each other. While learning the nodule area, we can notice the impact of different density types, which can help the model further improve the recognition accuracy of the two tasks

### 2.4. Test Process

For the detection and qualitative diagnosis of pulmonary nodules by the imaging physician group, a senior resident shall first detect the nodules on the high-resolution thin-layer chest CT images and diagnose the benign possible or suspicious malignant nodes according to the size, density, shape, and relationship with the surrounding blood vessels and bronchus and then complete the examination by the deputy chief physician. The other two imaging physicians with senior professional titles combined with artificial intelligence and referred to the reviewed image report for nodule detection and identification. When they disagree, they combined with multiplanar reconstruction and discussed to obtain consistent results, which will be used as the gold standard for true nodule detection. The gold standard for diagnosing benign and malignant pulmonary nodules was the postoperative pathological results. The density, size, benign, and malignant of each nodule were recorded, respectively. The nodule was divided into solid nodule and ground glass nodule. In order to further explore the effect of deep learning model on contour segmentation, the maximum cross-sectional diameter of nodules is divided to obtain the effect of the model under different sizes of nodules. The size of the nodule was divided into diameter <3 mm and ≥3 mm.

### 2.5. Evaluation Index of Classification and Segmentation of Pulmonary Nodules

The average CT density classification accuracy index was used for pulmonary nodule density classification, and the average Dice coefficient of each pulmonary nodule was used for pulmonary nodule segmentation. The calculation formula of the Dice coefficient is as follows:

(1) $$\begin{array}{c} \text{Dice}=\frac{2\times \left|\text{AI}\cap \text{Doc}\right|}{\left|\text{AI}\right|+\left|\text{Doc}\right|}, \end{array}$$

where |AI∩Doc| represents the overlapping area between the system model segmentation and the gold standard and |AI| + |Doc| represents the sum of the nodule area segmented by the model and the corresponding nodule area in the gold standard. When the result of model segmentation is consistent with the related consequence in the gold standard, the Dice coefficient is 1; when the two do not overlap, the Dice coefficient is 0.

### 2.6. Statistical Processing

In this study, SPSS 22.0 statistical software package was used for data analysis and processing; the accuracy of pulmonary nodule density classification and the Dice coefficient of segmentation were counted by SciPy 1.4.1 software. The accuracy of age and density classification and Dice coefficient conform to the normal distribution, expressed in $\bar{x}\pm s\;$; rate and frequency were used to describe the number of nodules. Analysis of variance was used to compare the classification accuracy and segmentation Dice coefficient of pulmonary nodules among three groups of different CT reconstruction algorithms. Inspection level *α* = 0.05.

## 3. Result

### 3.1. Classification Results of Pulmonary Nodule Density Types under Three CT Reconstruction Algorithms

Under three different CT reconstruction algorithms, the classification accuracy of 55 CT nodules and the classification accuracy of solid and subsolid nodules were higher (Table 1). The difference was not statistically significant (*P* > 0.05).

### 3.2. Segmentation Results of Model Pulmonary Nodules under Three CT Reconstruction Algorithms

For lung reconstruction, mediastinal reconstruction, and bone reconstruction, there was no significant difference in Dice coefficients of all nodules, solid nodules and subsolid nodules under the three different reconstruction algorithms (all *P* > 0.05) (Table 2).

Under three different CT reconstruction algorithms, the Dice coefficient increased with the increase of the diameter of pulmonary nodules (Figure 2).

### 3.3. Results of Benign and Malignant Diagnosis of Model Pulmonary Nodules under Three CT Reconstruction Algorithms

From the postoperative pathological results, there were 29 cases of malignant pulmonary nodules (Figure 3) and 26 cases of benign pulmonary nodules (Figure 4). The results of three reconstruction algorithms for identifying benign and malignant pulmonary nodules are shown in Table 3. There was no significant difference of accuracy between benign and malignant pulmonary nodules under different reconstruction algorithms (*P* > 0.05).

## 4. Discussion

The early imaging signs of lung cancer are primarily pulmonary nodules. At present, the clinical diagnosis and evaluation of pulmonary nodules are generally through clinical data, imaging data, tumor markers, pathological biopsy, surgical treatment, etc. It is common to screen and diagnose pulmonary nodules by imaging methods [17, 18]. The chest plain CT images can clearly distinguish and judge pulmonary nodules' size, position, morphology, and internal characteristics [19]. It is of great significance to distinguish the clinic's benign and malignant pulmonary nodules. Under different CT reconstruction algorithms, doctors' diagnoses vary widely. Thus, it is essential to observe the impact of images under different CT reconstruction algorithms on benign and malignant pulmonary nodule models and doctors' diagnoses [20–22]. The image in mediastinal reconstruction is smooth, the image in bone window reconstruction is sharp, and the image in lung window reconstruction is between the two. Different window reconstructions can diagnose various related diseases [23, 24].

In order to solve the instability of automatic segmentation of pulmonary nodules and classification of nodule density types under different CT reconstruction algorithms, a deep neural network model based on joint learning of pulmonary nodule segmentation and density type classification is proposed, which makes full use of the complementarity between the two tasks to promote each other [25]. At the same time, the model innovatively integrates many technologies such as a 3D convolution network, attention mechanism, and recurrent neural network to ensure that the model can thoroughly learn the local and global features of pulmonary nodules [26, 27]. The new method can carry out effective feature fusion to enhance the expression ability of the extracted features to improve the model's effectiveness for feature extraction under different image quality.

The test results of 55 pulmonary nodules in this study showed no significant difference in the classification accuracy of pulmonary nodules under different reconstruction algorithms (*P* > 0.05). There was no significant difference in the Dice coefficient of nodule segmentation under different reconstruction algorithms (*P* > 0.05). The model was stable under different CT reconstruction algorithms. The statistical results of pulmonary nodules grouped according to different sizes also show that the model effect improves with the increase of nodules. Except for nodules below 3 mm, the segmentation effect of the same group is stable under different reconstruction algorithms. The contours of benign and malignant nodules segmented by the model under different reconstruction algorithms are very similar, maintaining high consistency, and the difference is not statistically significant (*P* > 0.05). In addition, by analyzing the effect of models with different sizes of nodules, it is found that the poor segmentation effect is mainly concentrated on the micronodules with diameters less than 3 mm. The size of micronodules is small, and the boundary is not easy to determine, resulting in the deviation of the Dice coefficient index. However, with the increase of nodules, the effect of the model continues to improve, and the clinical analysis of larger nodules is of greater significance, indicating that the model meets the clinical needs. For the benign and malignant nodules, the models with different reconstruction algorithms had high sensitivity in diagnosing benign and malignant pulmonary nodules, and the difference was not statistically significant (*P* > 0.05).

## 5. Conclusions

In conclusion, the model constructed in this paper shows good performance in pulmonary nodule segmentation and density type classification and is stable under different CT reconstruction algorithms and has good diagnostic efficiency for benign and malignant pulmonary nodules, which shows that it has certain practical value in clinic. Due to the small scale of cases, this method has less classification of subsolid nodules and lacks certain validation. Future research can add data to verify the effectiveness of the model.

## Figures and Tables

**Figure 1:** Model framework of pulmonary nodule density type classification and contour segmentation based on deep learning.

**Figure 2:** Dice coefficient in different diameter of pulmonary nodules.

**Figure 3:** Segmentation of malignant pulmonary nodules under three reconstruction algorithms. (a) Lung window reconstruction. (b) Mediastinal reconstruction. (c) Bone window reconstruction.

**Figure 4:** Segmentation of benign pulmonary nodules under three reconstruction algorithms. (a) Lung window reconstruction. (b) Mediastinal reconstruction. (c) Bone window reconstruction.

**Table 1:** Accuracy analysis of 55 pulmonary nodules density types under three different reconstruction algorithms (*n*/%).

Reconstruction algorithm	All nodules (*n* = 55)	Solid nodule (*n* = 39)	Subsolid nodule (*n* = 16)
Lung window	54/98.2	38/97.4	16/100.0
Mediastinal window	53/96.4	38/97.4	15/93.8
Bone window	52/94.5	37/94.9	15/93.8
*χ* ^2^ value	1.038	0.518	1.043
*P* value	0.595	0.772	0.593

**Table 2:** segmentation results of 55 pulmonary nodules under three different reconstruction algorithms (Dice coefficient) (%).

Reconstruction algorithm	All nodules (*n* = 55)	Solid nodule (*n* = 39)	Subsolid nodule (*n* = 16)
Lung window	80.32 ± 5.91	79.93 ± 5.74	82.62 ± 6.28
Mediastinal window	79.83 ± 6.12	79.28 ± 5.39	82.35 ± 6.49
Bone window	80.17 ± 5.89	80.05 ± 6.21	81.79 ± 6.56
*F* value	1.683	1.590	1.753
*P* value	0.281	0.237	0.315

**Table 3:** Diagnostic accuracy under three different reconstruction algorithms (%).

Reconstruction algorithm	Sensitivity	Specificity	Accuracy
Lung window	96.6	100.0	98.2
Mediastinal window	93.1	100.0	96.4
Bone window	93.1	96.1	94.5
*χ* ^2^ value	0.424	2.026	1.038
*P* value	0.809	0.363	0.595

## Data Availability

The data used to support the findings of this study are available from the corresponding author upon request.
